The article "Correlation between Lpa, APO-A, APO-B, and Stenosis of Middle Cerebral Artery in Patients with Cerebral Ischemic Stroke" was retracted in 2023. Reasons: signs of a paper mill; suspected computer-generated content; unreliable results or conclusions; lack of ethics approval or compliance.

# Correlation between Lpa, APO-A, APO-B, and Stenosis of Middle Cerebral Artery in Patients with Cerebral Ischemic Stroke

**DOI:** 10.1155/2022/6403645

**Published:** 2022-11-14

**Authors:** Xinxu Chen, Xuefei Lu, Wei Li, Hongyan Zhang, Tan Wang

**Affiliations:** ^1^Department of Neurology, The First Affiliated Hospital of Hainan Medical University, Haikou, Hainan 570102, China; ^2^Department of Anesthesiology, The First Affiliated Hospital of Hainan Medical University, Haikou, Hainan 570102, China

## Abstract

Ischemic stroke (CIS) is characterized by a high incidence, disability, and mortality. Numerous studies have demonstrated that intracranial arterial stenosis is an important pathological basis of CIS, and its main cause is atherosclerosis. Dyslipidemia is an important risk factor for atherosclerosis. Lysophosphatidic acid (Lpa), apolipoprotein -A(APO-A), and apolipoprotein -B(APO-B) proved to be significantly correlated with the severity of coronary artery disease. This study retrospectively collected the case data of 186 patients with CIS treated from May 2020 to May 2022 and explored the correlation between Lpa, APO-A, APO-B, and middle cerebral artery (MCA) stenosis in CIS patients.

## 1. Introduction

Cerebral ischemic stroke (CIS) is the most common type of cerebrovascular disease, accounting for about 70% of all acute cerebrovascular diseases, with high morbidity, mortality, and recurrence rates [1]. Neurological deficits are a major feature of CIS, and symptoms associated with neurological deficits can generally peak in seconds or minutes due to the rapid onset of the disease. Occlusion of the middle cerebral artery (MCA) is one of the main causes of CIS and also the cause of patients, disorders of consciousness, cerebral edema, cerebral hernia, and even death [2]. At present, it is considered that atherosclerosis is the primary factor of MCA occlusion, and dyslipidemia is an important risk factor for atherosclerosis [3]. Lysophosphatidic acid (Lpa) is a kind of phospholipid, which is an intermediate product of glycerophospholipid metabolism [4]. Apolipoprotein (APO) is an apolipoprotein in the blood where the main function is to transport blood lipids to various tissues of the body and participate in the occurrence and regulation of cardiovascular and cerebrovascular diseases [5]. APO-A and APO-B are members of the APO family. Among them, APO-A is the main structural protein of high-density lipoprotein, and its main role is to remove tissue lipids and resist atherosclerosis. APO-B mainly exists on the surface of low-density lipoprotein, which can directly reflect the level of low-density lipoprotein cholesterol [6]. Some studies have shown that the development of atherosclerosis is also closely related to the metabolic process of APO-A and APO-B. In addition, previous studies [7, 8] have reported that Lpa, APO-A, and APO-B are significantly correlated with the severity of coronary artery disease. However, there are few reports about the correlation between Lpa, APO-A, and APO-B and the degree of cerebral artery stenosis Based on this, this study intends to retrospectively analyze the correlation between Lpa, APO-A, APO-B, and MCA stenosis in CIS patients, aiming to provide a new research direction for clinical prevention and treatment of CIS.

The article "Correlation between Lpa, APO-A, APO-B, and Stenosis of Middle Cerebral Artery in Patients with Cerebral Ischemic Stroke" was retracted in 2023. Reasons: signs of a paper mill; suspected computer-generated content; unreliable results or conclusions; lack of ethics approval or compliance.

## 2. Materials and Methods

### 2.1. General Information

The case data of 186 CIS patients admitted to our hospital from May 2020 to May 2022 were retrospectively selected for research. According to the DSA evaluation results, they have been divided into 92 cases without MCA stenosis group and 94 cases in the MCA stenosis group, including 18 cases, 16 cases, and 60 cases of mild, moderate, and severe MCA stenosis.

Inclusion criteria is as follows: (1) imaging examinations and clinical signs of all patients met the relevant diagnostic criteria of CIS [9]; (2) clinical data were complete, and research and analysis were available. Exclusion criteria is as follows: (1) Hemorrhagic stroke or cerebral thrombosis caused by other causes; (2) diseases affecting blood lipid levels other than conventional chronic underlying diseases, including coronary heart disease, diabetes, and hyperlipidemia; (3) take within one month before admission lipid-lowering drug treatment; and (4) there is a malignant tumor. This study is a retrospective study and does not involve ethical issues.

### 2.2. Data Collection

According to the purpose of this study, hospital professionals collected the age, gender, underlying diseases, smoking history, drinking history, systolic blood pressure (SBP), diastolic blood pressure (DBP), and the level of glycosylated hemoglobin (HbA1c), homocysteine (Hcy), uric acid level, and other data of the patient through the hospital medical record system. Wherein the underlying diseases include hyperlipidemia, type 2 diabetes mellitus, and coronary heart disease.

### 2.3. Middle Cerebral Artery Stenosis Assessment

All patients with CIS admitted to the hospital were evaluated for stenosis by digital subtraction angiography (DSA) using Aginnova digital subtraction X-ray angiography machine (model: Innova 3100-IQ) by the same group of physicians. Intracranial artery stenosis degree = (1 − diameter at the most stenotic point/diameter of the artery distal to the stenosis) × 100%. Classification of cerebral artery stenosis: less than 50% stenosis is mild, 50% to 69% is moderate, and more than 70% is severe [10].

The article "Correlation between Lpa, APO-A, APO-B, and Stenosis of Middle Cerebral Artery in Patients with Cerebral Ischemic Stroke" was retracted in 2023. Reasons: signs of a paper mill; suspected computer-generated content; unreliable results or conclusions; lack of ethics approval or compliance.

### 2.4. Method for Detecting Lpa, APO-A, and APO-B Levels

Within 48 h after hospitalization, 2 ml venous blood was collected from the upper limbs in the fasting state in the morning. The levels of total cholesterol (CHOL), triglyceride (TG), high-density lipoprotein (HDL), and low-density lipoprotein (LDL) were measured by Mindray BS2000 automatic biochemical analyzer. The levels of Lpa, APO-A, and APO-B were detected by an immunoturbidimetric kit (Wuhan Boster Biological Engineering Co., Ltd.), and the ratio of APO-A/APO-B was calculated.

### 2.5. Statistical Methods

SPSS 22.0 statistical software was used for data analysis, and the measurement data that met the normal distribution were expressed as (±*S*), and the differences between the two groups were compared by independent samples *t*-test. Differences between multiple groups were compared by one-way analysis of variance; measurement data that did not meet the normal distribution were expressed by M(P25, P75), and differences between groups were compared by Kruskal–Wallis test. The enumeration data were expressed by the number of cases and the rate, and the differences between groups were compared by the *χ*^2^ test. Logistic regression was used to analyze the independent risk factors of MCA stenosis. ROC was used to detect the diagnostic value of each index, and the Delong Test function was used to compare the AUC between the ROC curves. *P* < 0.05 indicates statistical significance.

## 3. Results

### 3.1. Comparison of Case Data between MCA Stenosis Group and No MCA Stenosis Group

There was no significant difference in gender, age, smoking, drinking, Hcy value, uric acid value, 24 hSBP value, and 24 hDBP value between the two groups (*P* > 0.05). The proportion of patients with hyperlipidemia, type 2 diabetes mellitus, and coronary heart disease in the MCA stenosis group was higher than that in the non-MCA stenosis group, and the HbA1c value was higher than that in the non-MCA stenosis group, and the differences were statistically significant (*P* < 0.05), as shown in Table 1.

### 3.2. Comparison of Blood Lipid Metabolism Indexes between MCA Stenosis Group and Non-MCA Stenosis Group

There was no significant difference in the levels of CHOL, TG, HDL, and LDL between the two groups (*P* > 0.05). The levels of Lpa and APO-B in the MCA stenosis group were higher than those in the non-MCA stenosis group, and the levels of APO-A, APO-A/APO-B were lower than those in the MCA stenosis group, and the differences were statistically significant (*P* < 0.05), as shown in Table 2.

### 3.3. Independent Influencing Factors of MCA Stenosis

Logistic regression analysis was performed with variables with statistical differences in Tables 1 and 2 as independent variables and MCA stenosis as dependent variables. The results showed that complicated with hyperlipidemia and coronary heart disease, high levels of Lpa and APO-B were independent risk factors for MCA stenosis in CIS patients (*P* < 0.05), and high levels of APO-A and APO-A/APO-B were independent protective factors (*P* < 0.05), as shown in Table 3.

The article "Correlation between Lpa, APO-A, APO-B, and Stenosis of Middle Cerebral Artery in Patients with Cerebral Ischemic Stroke" was retracted in 2023. Reasons: signs of a paper mill; suspected computer-generated content; unreliable results or conclusions; lack of ethics approval or compliance.

### 3.4. The Diagnostic Value of Lpa, APO-A, and APO-B in MCA Stenosis in CIS Patients

The results of the ROC curve showed that the AUCs of Lpa, APO-A, and APO-B alone and in combination were 0.647, 0.660, 0.672, and 0.762, respectively, and the diagnostic value of combined detection was higher than that of each index alone (*P*=0.014, 0.004, 0.003), as shown in Figure 1 and Table 4.

### 3.5. Comparison of Lpa, APO-A, and APO-B in CIS Patients with Different Degrees of MCA Stenosis

There were significant differences in the levels of Lpa, APO-A, and APO-B in CIS patients with different degrees of MCA stenosis (*P* < 0.05), as shown in Table 5.

### 3.6. Correlation Analysis of Lpa, APO-A, APO-B Levels in Peripheral Blood and Stenosis Degree of MCA in CIS Patients

The results of Spearman correlation analysis showed that the levels of Lpa and APO-B in the peripheral blood of CIS patients were positively correlated with the degree of MCA stenosis (*r* = 0.244, 0.286, *P* < 0.05). APO-A level was negatively correlated with the degree of MCA stenosis (*r* = −0.344, *P* < 0.001). The distribution of Lpa, APO-A, and APO-B levels in CIS patients with different degrees of MCA stenosis is shown in Figure 2, and the correlation between Lpa, APO-A, and APO-B and the degree of MCA stenosis is shown in Figure 3.

## 4. Discussions

MCA stenosis is a common type of intracranial arterial stenosis. According to statistics, intracranial artery stenosis may have a probability of 30%–50% of CIS, and MCA stenosis is one of the main pathological basis of CIS [11]. MCA is the main branch of the internal carotid artery, which controls the blood circulation in brain regions and is related to the movement, sensation, and language of the human body. Therefore, CIS caused by MCA stenosis may lead to hemiplegia and aphasia among other serious sequelae. In the study of Han et al. [12], 562 young patients with CIS were studied, and 249 CIS patients had MCA stenosis, accounting for 44.31%. In this study, DSA evaluation was performed on 186 patients with CIS, and 94 patients were found to have MCA stenosis, accounting for 50.54%, which was comparable to the above reports. It further confirms the prevalence of MCA stenosis in patients with CIS. This also suggests that early detection and control of risk factors affecting MCA stenosis have important clinical significance for preventing the occurrence and development of CIS.

The article "Correlation between Lpa, APO-A, APO-B, and Stenosis of Middle Cerebral Artery in Patients with Cerebral Ischemic Stroke" was retracted in 2023. Reasons: signs of a paper mill; suspected computer-generated content; unreliable results or conclusions; lack of ethics approval or compliance.

In this study, Logistic regression analysis showed that hyperlipidemia and coronary heart disease were independent risk factors for MCA stenosis in CIS patients (*P* < 0.05). A number of studies have shown that hyperlipidemia and coronary heart disease are independent risk factors for MCA stenosis [13, 14]. Hyperlipidemia is often accompanied by dyslipidemia in organisms, and lipids are deposited in large amounts in blood vessels, which gradually leads to atherosclerosis. As the intima of the cerebral artery thickens, it gradually leads to the narrowing of the MCA. Although coronary heart disease is a typical heart disease, a larger thrombus will be formed after the disease develops to a certain extent. As the blood circulates into different arteries, it is most likely to enter the MCA and then develop into MCA stenosis. It is therefore recommended that for patients with thrombus diseases such as hyperlipidemia and coronary heart disease, timely reduce the blood lipid level of the patient, improve the unhealthy state of the body with high load, adjust the diet balance, and take medicine strictly according to the doctor's advice.

This study showed that the levels of Lpa and APO-B in the MCA stenosis group were higher than those in the nonstenosis group, and the levels of APO-A and APO-A/APO-B were lower than those in the stenosis group (*P* < 0.05). Lpa, APO-A, and APO-B are closely related to MCA stenosis. Lpa is a bioactive phospholipid mediator that can induce cell proliferation and morphological changes, promote platelet aggregation, and form thrombosis [15]. The study by Chi et al. [16] reported that Lpa could damage the blood-brain barrier and lead to an increase in cerebral infarction volume. Bhattarai et al. [17] found in their mouse study that blocking the automatic axis protein (ATX)-Lpa signal could reduce the damage to the blood-brain barrier and mitochondrial function after blood reperfusion. The results of this study, combined with the above reports confirmed that Lpa was closely related to the formation of MCA stenosis and plaque stability in CIS patients. APO is a type of protein that can bind to plasma lipids (mainly triglycerides, cholesterol, and phospholipids) and also plays an important role in the occurrence and development of atherosclerosis [18]. Li et al. [19] studied the relationship between APO-A1, APO-B, and CIS patients with extracranial artery stenosis and found that APO-A1 and APO-B were closely related to intracranial artery stenosis. The study by Chou et al. [20] found that APO-B was a significant risk predictor of stroke. And Emanuele et al. [21] found that APO-A may be associated with poststroke dementia. Combined with the above reports, this study suggests that APO-A and APO-B may be the influencing factors of MCA stenosis in CIS patients.

The article "Correlation between Lpa, APO-A, APO-B, and Stenosis of Middle Cerebral Artery in Patients with Cerebral Ischemic Stroke" was retracted in 2023. Reasons: signs of a paper mill; suspected computer-generated content; unreliable results or conclusions; lack of ethics approval or compliance.

The ROC curve results for the Lpa, APO-A, and APO-B indices in this study showed AUC values of 0.647, 0.660, 0.672, and 0.762, respectively, both individually and in combination. The diagnostic value of the combined detection was higher than that of single indicators. These results indicated that each index had a certain diagnostic value for MCA stenosis in CIS patients, and the combined detection of the three indexes has a higher diagnostic value. The relationship between Lpa, APO-A, APO-B, and MCA stenosis was further analyzed using the Spearman correlation. The results showed that the levels of Lpa and APO-B in CIS patients were positively correlated with the degree of MCA stenosis, and the APO-A level was negatively correlated with the degree of MCA stenosis. It has been reported by Shui et al. [22] that the increase in Lpa is positively correlated with the progression of coronary artery disease. Yaseen et al. [23] reported that APO-B was positively correlated with the degree of coronary artery disease. In this study, combined with the above reports, it is suggested that when the levels of Lpa and APO-B are increased and the level of APO-A is decreased, the risk of MCA stenosis increases.

In conclusion, the levels of Lpa, APO-A, and APO-B in the peripheral blood of CIS patients have a certain correlation with the degree of MCA stenosis. When the levels of Lpa and APO-B increase and the level of APO-A decreases, the risk of MCA stenosis occurs. However, there are still some deficiencies in this study. If it is a retrospective study, there may be some data bias, and the specific mechanism of action of each index has not been clarified. In the later stage, further in-vitro animal experiments are still needed for in-depth research.

## Figures and Tables

**Figure 1:** The ROC curve of Lpa, APO-A, and APO-B in the diagnosis of MCA stenosis in CIS patients.

**Figure 2:** Distribution of Lpa, APO-A, and APO-B levels in CIS patients with different degrees of MCA stenosis. (a) Mild MCA stenosis. (b) Moderate MCA stenosis. (c) Severe MCA stenosis.

**Figure 3:** Scatter plot of correlation between Lpa, APO-A, APO-B, and MCA stenosis degree in CIS patients.

**Table 1:** Comparison of case data between the MCA stenosis group and the no MCA stenosis group.

Indexes	MCA stricture group (*n* = 94)	Non-MCA stricture group (*n* = 92)	*χ*2 value or *Z* value or *t* value	*P* value
Male [*n* (%)]	64 (68.09)	65 (70.65)	0.144	0.704
Age ($\bar{x}$ ± *s*, years)	60.14 ± 13.11	59.59 ± 12.07	0.298	0.766
Hyperlipidemia [*n* (%)]	51 (54.26)	18 (19.57)	23.978	<0.001
Type 2 diabetes [*n* (%)]	24 (25.53)	12 (13.04)	4.646	0.031
Coronary heart disease [*n* (%)]	15 (15.96)	4 (4.35)	6.833	0.009
Smoking [*n* (%)]	41 (43.62)	34 (36.96)	0.857	0.355
Drinking [*n* (%)]	27 (28.72)	26 (28.26)	0.005	0.944
HbA1c [M(P_25_, P_75_), %]	6.00 (5.70, 6.63)	5.80 (5.60, 6.28)	−2.299	0.021
Hcy [M(P_25_,P_75_), *μ*mol/L]	8.80 (5.01, 13.00)	8.34 (6.86, 12.19)	0.323	0.747
Uric acid ($\bar{x}$ ± *s*, *μ*mol/L)	294.43 ± 73.41	321.50 ± 72.53	1.880	0.062
24 hSBP ($\bar{x}$ ± *s*, mmHg)	139.76 ± 17.71	137.63 ± 19.30	0.783	0.435
24 hDBP ($\bar{x}$ ± *s*, mmHg)	81.88 ± 10.52	81.70 ± 11.28	0.117	0.907

The article "Correlation between Lpa, APO-A, APO-B, and Stenosis of Middle Cerebral Artery in Patients with Cerebral Ischemic Stroke" was retracted in 2023. Reasons: signs of a paper mill; suspected computer-generated content; unreliable results or conclusions; lack of ethics approval or compliance.

**Table 2:** Comparison of blood lipid metabolism indexes between the MCA stenosis group and the no MCA stenosis group.

Indexes	MCA stricture group (*n* = 94)	Non-MCA stricture group (*n* = 92)	*Z* value or *t* value	*P* value
Lpa [M(P_25_,P_75_), mg/L]	193.14 (154.82, 363.85)	135.63 (78.01, 326.22)	3.472	0.001
CHOL ($\bar{x}$ ± *s*, mmol/L)	4.75 ± 1.23	4.82 ± 1.10	0.451	0.653
TG [M(P_25_, P_75_), mmol/L)	1.35 (1.05, 1.68)	1.25 (0.89, 1.74)	1.219	0.223
HDL [M(P_25_, P_75_), mmol/L]	1.22 (0.93, 1.44)	1.21 (0.99, 1.44)	0.706	0.480
LDL ($\bar{x}$ ± *s*, mmol/L)	2.87 ± 0.68	2.95 ± 0.67	0.591	0.556
APO-A [M(P_25_, P_75_), g/L]	1.11 (1.00, 1.29)	1.22 (1.07, 1.39)	2.917	0.004
APO-B ($\bar{x}$ ± *s*, g/L)	1.02 ± 0.29	0.94 ± 0.25	2.390	0.018
APO-A/APO-B [M(P_25_, P_75_)]	1.12 (0.87, 1.39)	1.32 (1.04, 1.70)	3.550	<0.001

**Table 3:** Independent influencing factors of MCA stenosis.

Indexes	B	Se	Wals	Exp (B)	95% confidence interval	*P*
Hyperlipidemia	−1.462	0.366	15.970	0.232	0.113–0.475	<0.001
Type 2 diabetes	−0.980	0.562	3.042	0.375	0.125–1.129	0.081
Coronary heart disease	−1.741	0.629	7.665	0.175	0.051–0.601	0.006
HbA1c	−0.102	0.159	0.409	0.903	0.661–1.234	0.522
Lpa	−1.001	0.401	6.231	2.721	1.240–5.971	0.013
APO-A	1.369	0.433	9.996	3.931	1.983–9.186	0.002
APO-B	−1.134	0.382	8.813	3.108	1.470–6.571	0.003
APO-A/APO-B	1.040	0.381	7.451	2.829	1.241–5.970	0.007

**Table 4:** The diagnostic value of Lpa, APO-A, and APO-B for MCA stenosis in CIS patients.

Indexes	AUC	Sensitivity (%)	Specificity (%)	95% confidence interval	*P*
Lpa	0.647	80.85	55.43	0.574∼0.716	<0.001
APO-A	0.660	70.21	54.35	0.587∼0.727	<0.001
APO-B	0.672	74.47	53.26	0.599∼0.739	<0.001
Joint detection	0.762	62.77	75.00	0.694∼0.821	<0.001

**Table 5:** Comparison of Lpa, APO-A, and APO-B in CIS patients with different degrees of MCA stenosis.

Degree of MCA stenosis	Lpa [M(P_25_, P_75_), mg/L]	APO-A [M(P_25_, P_75_), g/L]	APO-B ($\bar{x}$ ± *s*, g/L)
Mild (*n* = 18)	165.93 (90.50, 254.51)	1.23 (1.05, 1.68)	0.90 ± 0.22
Moderate (*n* = 16)	213.00 (157.29, 353.25)	1.17 (1.05, 1.32)	0.96 ± 0.27
Severe (*n* = 60)	262.00 (163.30, 417.75)	1.09 (0.93, 1.21)	1.10 ± 0.30
*Z*/*F*	6.565	7.057	4.191
*P*	0.038	0.029	0.018

The article "Correlation between Lpa, APO-A, APO-B, and Stenosis of Middle Cerebral Artery in Patients with Cerebral Ischemic Stroke" was retracted in 2023. Reasons: signs of a paper mill; suspected computer-generated content; unreliable results or conclusions; lack of ethics approval or compliance.

## Data Availability

The data used and/or analyzed during the current study are available from the corresponding author.
